# Role of ABCB1 in mediating chemoresistance of triple-negative breast cancers

**DOI:** 10.1042/BSR20204092

**Published:** 2021-02-17

**Authors:** Yomna S. Abd El-Aziz, Andrew J. Spillane, Patric J. Jansson, Sumit Sahni

**Affiliations:** 1 Northern Clinical School, Faculty of Medicine and Health, University of Sydney, NSW, Australia; 2 Kolling Institute of Medical Research, St Leonards, NSW, Australia; 3 Oral Pathology Department, Faculty of Dentistry, Tanta University, Tanta, Egypt; 4 Melanoma Institute Australia, University of Sydney, Wollstonecraft, NSW, Australia; 5 Northern Sydney Cancer Centre, Royal North Shore Hospital, St Leonards, NSW, Australia; 6 Cancer Drug Resistance Program, University of Sydney, Sydney, New South Wales 2006, Australia

**Keywords:** breast cancers, multidrug resistance, p-glycoprotein, triple negative breast cancer

## Abstract

Triple-negative breast cancer (TNBC) is a group of breast cancers which neither express hormonal receptors nor human epidermal growth factor receptor. Hence, there is a lack of currently known targeted therapies and the only available line of systemic treatment option is chemotherapy or more recently immune therapy. However, in patients with relapsed disease after adjuvant or neoadjuvant therapy, resistance to chemotherapeutic agents has often developed, which results in poor treatment response. Multidrug resistance (MDR) has emerged as an important mechanism by which TNBCs mediate drug resistance and occurs primarily due to overexpression of ATP-binding cassette (ABC) transporter proteins such as P-glycoprotein (Pgp). Pgp overexpression had been linked to poor outcome, reduced survival rates and chemoresistance in patients. The aim of this mini-review is to provide a topical overview of the recent studies and to generate further interest in this critical research area, with the aim to develop an effective and safe approach for overcoming Pgp-mediated chemoresistance in TNBC.

## Triple-negative breast cancer

Breast cancer is the most common cause of cancer-related deaths in women [1]. It is a heterogeneous group of cancers currently most commonly categorized into four main types according to immunohistochemical profile and increasingly confirmed by gene expression profile testing: (**1**) Luminal A which is positive for estrogen receptor (ER) and progesterone receptor (PR) and negative for epidermal growth factor receptor 2 (HER-2) receptor and low Ki67; (**2**) Luminal B which is positive for ER and sometimes HER-2 and low or negative for PR with a high Ki67; (**3**) HER-2 positive tumors that are HER-2 positive and negative for ER and PR; (**4**) triple-negative breast cancer (TNBC) which is negative for ER, PR, and HER-2 expression. TNBC accounts for approximately 15% of all breast cancers [2]. TNBCs are highly heterogeneous and have been further characterized into six subtypes, namely, basal-like 1 (BL1), basal-like 2 (BL2), an immunomodulatory (IM), a mesenchymal (M), a mesenchymal stem-like (MSL), and a luminal androgen receptor (LAR) subtype [3]. These TNBC subtypes have been shown to be independent predictor of pathological complete response (pCR) after neoadjuvant chemotherapy [4].

Due to molecular expression pattern, TNBC cannot be treated with hormonal or HER-2-targeted therapies and currently chemotherapy and increasingly immune therapy are the only available systemic therapeutic strategy for treatment. The most commonly used chemotherapeutic agents are taxanes (e.g., Paclitaxel), anthracyclins (e.g., Doxorubicin), and platinums (e.g., carboplatins) [5]. The patients are commonly recommended chemotherapy under neoadjuvant settings to decrease the size of the tumor before surgery, as well as under adjuvant and metastatic therapeutic settings. Approximately 50% of tumors have a pCR to neoadjuvant chemotherapy but up to 65% if Pembrolizumab is added [6]. Unfortunately, not all patients benefit from chemotherapy, as some cases exhibit metastatic relapse and either have primary or develop secondary drug resistance [7].

## Development of drug resistance

As cancer cells can undergo different mutations with time, cancer is often a ‘moving target’ that can adapt to overcome challenges and microenvironmental stressors they are enduring. One of these challenges is the anti-cancer agents, which the cancer cells try to evade by up-regulating resistance mechanisms against these drugs. Drug resistance can be defined as a decrease in drug’s ability to effectuate its action and can be manifested by local recurrence or metastasis most commonly within 5 years of primary TNBC treatment. The drug resistance may be due to intrinsic or acquired factors. Intrinsically derived drug resistance can be observed in tumors that exhibit poor initial response to chemotherapy without prior exposure to anti-cancer agents, while, the acquired type can be seen in tumors that demonstrates an initial good response to treatment followed by adaptation and resistance to the drug treatment, often resulting in a cancer type with a more aggressive behavior [8]. Intrinsic factors may be due to genomic instability of cancer cells which is responsible for intra-tumor heterogeneity [9]. This heterogeneity results in evolution of drug-resistant subclone [10]. The genomic instability can be in the form of point mutation, deletion, chromosomal translocation [11], or epigenetic changes such as DNA methylation [12]. The extrinsic factors include drug breakdown, modified expression of drug’s target, reduced drug absorption or increased release of the drug outside the cells [9].

Drug efflux pumps are known to play an important role in drug resistance. The drug transport depends on the activity of ATP-binding cassettes (ABC superfamily) which is membrane transporter proteins that pump the chemotherapeutic drug outside the cell. This prevents intracellular accumulation of drugs and eventually, decrease their efficacy resulting in resistance [13].

## ATP-binding cassettes (ABC superfamily)

ABC superfamily is a large, diverse group of membranous proteins that act as pumps to efflux substances out of the cell. These proteins depend on energy derived from ATP hydrolysis to transport different compounds against their electrochemical gradient across the cell membrane [14]. The compounds include amino acids, peptides, sugar, metal ions, metabolites, and hydrophobic compounds [15]. ABC superfamily, via its transporting property, control levels of lipids, hormones, and ions inside the cells and regulate many intracellular organelles such as lysosomes [16] and Golgi apparatus [17]. These pumps are also known to be involved in mediating chemotherapy resistance in cancer [15]. ABC superfamily comprises 48 proteins which are subdivided into seven subfamilies designated from ABC-A to ABC-G according to their sequence similarities [18]. P-glycoprotein (Pgp) is a member of ABC-B subfamily and is known to play a crucial role in mediating multidrug resistance (MDR) in cancer [19].

## Pgp or ABCB1 or MDR1

Pgp is a 170-kDa membranous protein that was first described by Ling et al*.* in 1976 as it was overexpressed in colchicine-resistant cell line [20]. Pgp is normally expressed in the epithelium of many different tissues such as blood–brain barrier, intestine, placenta and kidney. It is situated at the apical part of the cell, resulting in the translocation of substrate from the basolateral part to the apical part of the cell [21]. Consequently, Pgp helps to protect the brain from any toxins, drugs or substances that are present in the blood and that is essential as the brain is highly sensitive and critical organ [22]. In the placenta, Pgp acts as a functional barrier between the maternal and fetal circulation which efflux any drugs or toxins and prevents its passage to the developing fetus [23]. In the liver and the intestine, Pgp transfers any drugs or toxins from the blood to be excreted in the bile and the faeces [21]. Pgp can transport wide variety of substances including many cytotoxic anticancer drugs. This explains the cross-resistance property that is conferred to cancer cells due to its expression. Hence, the designation of ‘multidrug resistance’ (MDR) was applied [24].

### Structure of Pgp

Structurally, Pgp consists of four domain architecture, two cytoplasmic domains called nucleotide-binding domains (NBDs) and two transmembrane domains (TMDs) (Figure 1). The NBDs are the binding site for ATP and responsible for its hydrolysis via ATPase, thus, producing energy required for efflux of substances outside the cell regardless of the concentration gradient [25]. Also, NBDs contains Walker A and B motifs and signature motifs which participate in ATP hydrolysis and energy production [26]. TMDs are sites where the substrates are verified and transported [25]. Each TMD has a structural fold which consists of six transmembrane helices [27]. Also, it has a NH_2_– and COOH– termini that are located in the cytoplasm and the first extracellular loop is heavily N-glycosylated [28].

**Figure 1:** Pgp structure Pgp structure composes of two transmembrane domains (TMDs) and two cytoplasmic domains (NBDs) which are the sites for ATP hydrolysis. Each TMD consists of six helices. Pgp molecule has NH_2_– and COOH– termini within the cytoplasm.

### Mechanism of action

The exact mechanism by which Pgp transports substances is still not clear. Most widely accepted models hypothesize that Pgp is subjected to a series of conformational changes when bound to the substrate and these changes are catalyzed by ATP hydrolysis [29]. Transmembrane segments may go back and forth through a channel formed by other transmembrane segments transferring the substrate from inside the cell to extracellular space [30]. This model is supported by several experimental studies [31–35].

More recently, it was found that Pgp is not only localized to the plasma membrane but is also, present on intracellular organelles, specifically, lysosomes [36]. It was demonstrated that lysosomal Pgp can confer to MDR via a unique mechanism (Figure 2) [37]. As lysosomes are formed from endosomes, which are in turn formed as vesicles from invagination of plasma membrane, the lysosomal Pgp is functionally active [38]. However, invagination of the membrane results in the inversion of Pgp topology, enabling it to pump substrates into the lysosomes [37,39]. Yamagishi et al*.* [37] demonstrated that lysosomal Pgp is responsible for trapping of Pgp substrates within the lysosome, preventing the chemotherapeutic drug from reaching its target (e.g., nucleus). This is due to ionization of chemotherapeutic agents at lysosomal pH, which hinders their diffusion through the lysosomal membrane. Thus, lysosomes are considered to be the ‘drug safe house’ which is used by cancer cells to overcome the chemotherapy. Consequently, lysosomal Pgp, in addition to membrane Pgp, could be a promising target to overcome MDR.

**Figure 2:** Pgp confers MDR via a dual mechanism (**A**) Pgp localized on the plasma membrane protects the cell by effluxing substrates out of the cells. During endocytosis, which is further facilitated by the tumor microenvironmental stressors, the plasma membrane invaginates, which results in topical inversion of Pgp orientation in the membrane of early endosome. The endosomes then mature into lysosomes with Pgp on their membrane still being functional with its active sites facing the cytosol. When a Pgp substrate, such as Paclitaxel enters the cells, it is not only pumped out via plasma membrane Pgp, but also pumped into lysosomes via lysosomal Pgp. Weakly basic Pgp substrates (ex: paclitaxel) tends to get entrapped within the lysosome through their ionization at the lysosomal pH. This mechanism leads to inactivity of Pgp substrates which target other organelles in the cell such as nucleus for paclitaxel. (**B**) In contrast, lysosomal targeting agents such as DpC hijacks this resistance pathway to induce lysosomal damage, which results in potent anti-cancer activity.

### Pgp substrates

Pgp can transport a wide range of different substrates. All substrates have a common amphipathic feature, which allows the substrates to be inserted properly in the inner hemi-leaflet of the cell membrane, and then turned over to the outer hemi-leaflet. Pgp substrates are usually organic compounds and may contain aromatic group but some substrates are non-aromatic. They frequently are basic in nature; however, some acidic substrates can be transported [40].

Pgp substrates include analgesics such as asimadoline; anticancer drugs e.g., Vinca alkaloids (vinblastine, vincristine), Taxanes (paclitaxel, docetaxel) and Anthracyclines (doxorubicin, daunorubicin, epirubicin); HIV protease inhibitors e.g., Saquinavir, Ritonavir and Nelfinavir; H2-receptor antagonists e.g., Cimetidine; Anti-gout agents e.g., Colchicine; Antidiarrheal agents e.g., Loperamide; Calcium channel blockers e.g., Verapamil (poor substrate); Cardiac glycosides e.g., Digoxin; Immunosuppressive agents e.g., Cyclosporin A; Corticoids e.g., Hydrocortisone; Antibiotics e.g., Erythromycin and Diagnostic dyes e.g., Rhodamine 123 [24].

### Role of Pgp in TNBC chemoresistance

Multidrug resistance is defined as the resistance of cancer cells to broad variety of chemotherapeutic agents. MDR occurs due to multiple mechanisms: altered drug targets, metabolic modification and detoxification, inhibition of apoptosis pathways, decreased drug influx, increased drug efflux predominantly via ABC superfamily transporters, and elevated expression levels of these drug efflux pumps [41]. Pgp is one of ABC transporter family which is overexpressed in different types of cancer and its expression is considered to be a predictor of poor prognosis [42–44]. It was also found that Pgp expression is related to higher relapse rates, decreased survival rates and chemotherapy resistance [43–45]. Notably, increased Pgp expression was noted after conventional chemotherapy of different tumor types including TNBC [46,47].

Two studies by Kim et al*.* [48] and Zhang et al*.* [49] demonstrated significant increase in Pgp expression, by immunohistochemistry, after neoadjuvant chemotherapy treatment of breast cancer, which was markedly higher in patients with no pathological response. In another study, Pgp expression was up-regulated after preoperative chemotherapy of breast cancer patients and associated with lymph node metastasis [50]. In a similar manner, chemoresistant TNBC cell line, developed by the continued treatment of HCC1806 cells with paclitaxel, exhibited increased expression levels of Pgp compared with the parent cell line [51]. Furthermore, Epirubicin-resistant TNBC cell line, MDA-MB-231, exhibited high Pgp expression, with restoration of sensitivity to Epirubicin after Pgp suppression [52].

Interestingly, the cytotoxicity of proteasome inhibitors was increased when combined with Pgp inhibitors in MDA-MB-231 and this combination also enhanced inhibition of tumor cell proliferation [53]. Moreover, targeting of lysosomes via lysosomal inhibitors in MDA-MB-231 down-regulated Pgp levels and restored endoplasmic reticulum stress-dependent apoptosis through preventing the degradation of CAAT/enhancer binding protein (C/EBP)-β LiP [54]. In addition, curcumin solid lipid nanoparticles (SLNs) demonstrated higher efficacy in increasing the cytotoxicity of doxorubicin against Pgp expressing TNBC by lowering levels of reactive oxygen species (ROS) with reduced activation of Pgp promoter transcription [55]. Overall, these interesting *in vitro* studies indicate that Pgp can potentially be targeted to reverse and overcome the MDR in TNBCs. However, more detailed studies examining the role of Pgp in TNBC, especially in human and animal models, are required to comprehensively understand how this molecule mediates MDR in TNBCs.

### Targeting Pgp to overcome MDR in TNBCs

Different therapeutic strategies have been evolved through the last two decades to target Pgp (Table 1). These strategies are described in details below.

**Table 1:** Different therapeutic strategies to overcome Pgp-mediated MDR

Pgp targeting strategies		Examples
Pgp inhibitors	First generation	Verapamil, cyclosporin, tamoxifen
	Second generation	Dexverapamil, dexniguldipine, valspodar, biricodar
	Third generation	Tariquidar, zosuquidar, elacridar
Utiliazing Lysosomal Pgp		Dp44mT, DpC
Pgp antibodies		UIC2

#### Pgp inhibitors

In the last two decades, there has been increasing interest on how to reverse the MDR through inhibition of Pgp activity. These extensive studies resulted in identification of many different agents that can modulate the function of Pgp. These agents were divided into three generations.

##### First generation

It was first introduced by Chan et al. [56] who used cyclosporin in combination with chemotherapy for treatment of neuroblastoma and achieved high cure rates. This generation includes verapamil, cyclosporin, tamoxifen and other calmoduline antagonist which are substrates for Pgp. They act by competing with the cytotoxic drug for efflux by Pgp pump. Unfortunately, they had a low binding affinity for Pgp and required high doses to produce the required effect which led to undesired toxicity [57]. It was found that the required dose to inhibit the Pgp activity resulted in toxic cardiovascular effect in humans [58]. Also, these compounds are substrates of other drug transporters that result in unpredictable pharmacokinetic action in presence of chemotherapeutic agents. All these limitations led to the evolution of the second- and third-generation Pgp inhibitors [57,59].

##### Second generation

This generation includes dexverapamil, dexniguldipine, valspodar and biricodar which are less toxic and more potent than those of the first generation [57]. Their efficacy had been proved by numerous clinical trial studies on different types of cancer [60–65]. Their administration with the cytotoxic drugs resulted in the reversal of MDR [62]. Despite this, these agents had some characteristics that hampered their clinical utility. These compounds inhibit the metabolism of the chemotherapeutic drugs that led to toxicity which necessitated lowering of their dose in clinical trials [66]. Additionally, these Pgp inhibitors are also substrates for other drug transporters, which may reduce the ability of normal cells to protect themselves against the cytotoxic drug [57].

##### Third generation

Tariquidar, zosuquidar and elacridar are agents from the third generation [67,68]. They showed higher potency than those of the second generation as they do not interfere with the pharmacokinetics of the cytotoxic drugs. These modulators are also highly specific for Pgp, which minimizes their effect on normal tissue [69]. The most promising agent of the third generation is tariquidar which exhibited higher efficacy than first and second generations in terms of potency and duration of action [69–71]. Patel et al*.* showed that re-sensitization of resistant ovarian cell line to paclitaxel can be achieved by co-delivery of tariquidar and paclitaxel via loaded long circulating liposomes which result in reversal of MDR [72]. In a same manner, Rottenberg et al*.* demonstrated that resistance to PARP inhibitor in TNBCs can be reversed, *in vivo*, by co-administration of tariquidar with PARP inhibitor [73]. Notably, increased doxorubicin efficacy was observed in doxorubicin-resistant TNBC cell line (i.e., MDA-MB-231DX), when treated with tariquidar [74]. However, these agents showed unexpected toxicity in phase III clinical trials as the combination of tariquidar with paclitaxel was associated with too much toxicity, which led to termination of the trial [75]. Taken together, either new Pgp inhibitors or alternate Pgp targeting strategies are required to overcome Pgp-mediated MDR.

#### Utilizing lysosomal Pgp to overcome MDR

Recently, studies were directed to overcome MDR via targeting the lysosomal Pgp. Thiosemicarbazones (e.g., Dp44mT, DpC) are anti-cancer agents which demonstrated anti proliferative activity and a crucial role in overcoming MDR through affecting the lysosomal integrity [37,76–79]. Cancer cells have been shown to have elevated levels of copper that can be used by Dp44mT to cause lysosomal damage. Once Dp44mT is administered, it become protonated and entrapped inside the acidic environment of the lysosomes via lysosomal Pgp. Then, it forms a redox active copper complex within the lysosomes that generate ROS which, in turn, induce lysosomal membrane permeability and cathepsin release to initiate apoptosis (Figure 2) [80]. Seebacher et al*.* [78] demonstrated that synergy existed between both doxorubicin and Dp44mT in TNBC cell line (MDA-MB231) which is dependent on Pgp expression level and lysosomal permeability as Dp44mT helps to release doxorubicin from its entrapment within lysosome and reach the nucleus (its target) resulting in potent inhibition of cancer cell proliferation*.* Moreover, Al-Akra et al*.* [39] displayed that different tumor microenvironmental stressors up-regulate lysosomal Pgp in TNBC cell line (MDA-MB-231), via HIF-1α-dependent pathway, which hinders doxorubicin from reaching its target (i.e., nucleus). In contrast, increased levels of lysosomal Pgp facilitate the action of thiosemicarbazones which leads to apoptosis [39]. These data indicate that that Dp44mT can hijack the lysosomal Pgp that lead to accumulation of Dp44mT into lysosomes and induction of lysosomal damage and cytotoxicity, and thus, could offer a potential novel therapeutic opportunity to overcome Pgp-mediated MDR in TNBCs [81].

#### Pgp antibodies

Another promising strategy that can be used to inhibit Pgp is immunotherapy using antibodies against Pgp. Several monoclonal antibodies have been developed against Pgp [82]. UIC2 is an IgG2a mouse monoclonal antibody which is directed against epitopes in Pgp structure [83]. Mechetner et al*.* demonstrated that UIC2 can inhibit the pumping activity of Pgp and its inhibitory effect is equal to some Pgp inhibitors, such as verapamil, at its highest clinical concentration [82]. Another study [84] showed that UIC2 has the ability to bind only to 10–40% of cell surface Pgp, whilst, its ability to bind the rest increases in presence of Pgp substrates or modulators. The investigators found that *in vitro* combination of UIC2 with Cyclosporine, at ten-fold lower concentration than that used for Pgp inhibition, decreased the EC_50_ value of doxorubicin in KBV1 (Pgp+) cells to the same level of KB31 (Pgp−) cells [84]. These results were consistent with *in vivo* studies in immunodeficient mice, which showed a significant decrease in Pgp^+^ tumor weight when treated with a combination of doxorubicin and UIC2 compared with doxorubicin alone [84]. Although, this strategy appears to be promising, currently no studies using TNBC models have been performed to ascertain its utility in overcoming Pgp-mediated MDR in TNBCs.

## Conclusion

MDR is an obstacle in cancer chemotherapy especially in tumors which highly express ABC transporters (e.g., Pgp). Recently, several attempts have been investigated to overcome the MDR by targeting Pgp through different inhibitors in combination with conventional chemotherapeutic agents. Unfortunately, to date, Pgp inhibitors have not shown any promising results in the clinical trials. Alternative therapeutic strategies such as targeting lysosomal Pgp (e.g., thiosemicarbazone anti-cancer agents) or use of monoclonal anti-Pgp antibodies provide a promising opportunity to develop effective treatments to overcome MDR in TNBCs. Clearly, further research in this area is warranted to develop novel therapies targeting Pgp-mediated MDR in TNBC.

## Abbreviations

ABC: ATP-binding cassette
ER: Estrogen recpetor
HER-2: epidermal growth factor receptor 2
HIF-1α: hypoxia inducible factor -1α
MDR: multidrug resistance
NBD: nucleotide-binding domain
PARP: poly ADP ribose polymerase
pCR: pathological complete response
Pgp: P-glycoprotein
PR: progesterone receptor
ROS: reactive oxygen species
TMD: transmembrane domain
TNBC: triple-negative breast cancer
